The article "Some Study of Semigroups of h-Bi-Ideals of Semirings" was retracted in 2023. Reasons: suspected computer-generated content; unreliable results or conclusions; concerns about the data; concerns about the results or conclusions.

# Some Study of Semigroups of **h**-Bi-Ideals of Semirings

**DOI:** 10.1155/2021/9908175

**Published:** 2021-12-13

**Authors:** Rukhshanda Anjum, Fairouz Tchier, Zeeshan Saleem Mufti, Qin Xin, Syed Irfan Ali Shah, Yae Ulrich Gaba

**Affiliations:** ^1^Department of Mathematics and Statistics, The University Of Lahore, Lahore, Pakistan; ^2^Department of Mathematics, King Saud University, P.O. Box 22452, Riyadh 11495, Saudi Arabia; ^3^Faculty of Science and Technology, University of the Faroe Islands, Vestarabryggja 15, FO 100 Torshavn, Faroe Islands, Denmark; ^4^Quantum Leap Africa (QLA), AIMS Rwanda Centre, Remera Sector KN 3, Kigali, Rwanda

## Abstract

Semigroups are generalizations of groups and rings. In the semigroup theory, there are certain kinds of band decompositions which are useful in the study of the structure of semigroups. This research will open up new horizons in the field of mathematics by aiming to use semigroup of *h*-bi-ideal of semiring with semilattice additive reduct. With the course of this research, it will prove that subsemigroup, the set of all right *h*-bi-ideals, and set of all left *h*-bi-ideals are bands for *h*-regular semiring. Moreover, it will be demonstrated that if semigroup of all *h*-bi-ideals (*B*(*H*), ∗) is semilattice, then *H* is *h*-Clifford. This research will also explore the classification of minimal *h*-bi-ideal.

## 1. Introduction

Primary idea of semigroup and monoid is given by Wallis [1]. Wallis expressed that a set which satisfies the associative law under some binary operations is called semigroup, and a set which is semigroup with identity is called monoid. Several researchers work on semigroup theory like [2, 3]. [4] discusses the actual concept of group and commutative group, as well as other major points. Vandiver [5] discussed semiring and elucidates several main concepts. He believed that an algebraic structure is made up of a nonempty set that can be manipulated using the binary operations (+) and (·). Semirings play a significant role in geometry, but they also play a role in pure mathematics. Several ideas and results relating semiring have been presented by different researchers like [6, 7]. Semirings with additive inverse are studied by Karvellas Goodearl, Petrich, and Reutenauer [8–11]. In Applied Mathematics and Information Sciences, semirings have been established for solving the different problems. Semirings with commutative addition and zero element are also very necessary in theoretical computer science.

Ideals of semiring are used in structure theory and have a wide variety of applications like in [12, 13]. In [14], Gan and Jiang investigated the notion of an “ordered semiring containing 0,” as well as several other definitions such as the maximal ideal, ordered ideals, and the minimum ideal of an ordered semiring. In [15], Han and others explored ordered semiring. Ma and Zhan uses the principle of ideal in [16], but he used the *h*-ideals, a new class of ideals proposed by Iizuka [17]. Zhan and others use this particular class of ideals in their study [18–22] for a variety of purposes specific to their analysis.

The article "Some Study of Semigroups of h-Bi-Ideals of Semirings" was retracted in 2023. Reasons: suspected computer-generated content; unreliable results or conclusions; concerns about the data; concerns about the results or conclusions.

The concept of regular semirings was introduced by Von Neumann [23] and Bourne [24]. Von Neumann showed that the ring (*H*, ·) would also be regular if the semigroup is regular. Bourne showed that if ∀*t* ∈ *H*, there exists *h*_1_, *h*_2_ ∈ *H* such that *t* + *th*_1_*t* = *th*_2_*t*, then the semiring is regular.

It was in 1952 that Good and Hughes [25] first described the definition of a bi-ideal of semigroup. Lajos suggested the (*m*, *n*)-ideals in [26]. As a generalization of *k*-clifford semirings, Bhuniya introduced the left *k*-clifford semiring [27]. New research in semigroups and semirings is advancing day by day in different fields of asymptotics, control theory, biology, and medicine [28–31].

We compare a semigroup *B*(*H*) of *h*-bi-ideal whose additive reduct is a semilattice in this article. As an extension of the inscription of bi-ideals in semigroup, we introduce *h*-bi-ideal of a semiring. Further, we have shown that the *h*-bi-ideal semigroup *B*(*H*) elegantly illustrates different sectors of a semiring.

This research represents *h*-regular semiring along their *h*-ideals. We will define the different subclass of the *h*-regular semiring by their semigroup of *h*-bi-ideals. Also, we will show that *B*(*H*) = *ℛ*(*H*)*ℒ*(*H*) for *h*-regular semiring *H*. We will characterize a new class of semigroup of *h*-bi-ideals in *h*-Clifford semiring. Lastly, we will work on minimal *h*-ideal along their *h*-bi-ideals and will prove that *B*_*m*_(*H*) is a rectangular band. This article is arranged in such a way that after passing through introduction in Section 1, we will discuss basic definitions in Section 2. We will work on construction of semigroups of *h*-bi-ideals in *h*-regular semiring in Section 3, and Section 4 will consist of semigroup of *h*-bi-ideals in *h*-Clifford semiring, a discussion on semigroup of minimal *h*-bi-ideal. Then, we will conclude our research in the last.

## 2. Preliminaries

Semiring (*H*, +, ·) is an algebra with two binary operation + and · such that both the additive reduct (*H*, +) and the multiplicative reduct (*H*, ·) are semigroups and are subject to the following distributive laws:

(1) $$\begin{array}{c} a_{1}\left(a_{2}+a_{3}\right)=a_{1}a_{2}+a_{1}a_{3},\\ \left(a_{1}+a_{2}\right)a_{3}=a_{1}a_{3}+a_{2}a_{3},\;\forall a_{i}\in H. \end{array}$$

Let *M* is a nonempty subset of semiring *H*, then *M* is said to be a band if *M* is a semigroup, and every element of *M* is an idempotent one.

The article "Some Study of Semigroups of h-Bi-Ideals of Semirings" was retracted in 2023. Reasons: suspected computer-generated content; unreliable results or conclusions; concerns about the data; concerns about the results or conclusions.

A band which is commutative is called semilattice. Throughout this, except as otherwise specified, *H* is a semiring such that the additive reduct is a semilattice, and this class of all such semiring is denoted by *HL*^+^.

Let *L* be nonempty subset of semiring *H*, then *L* is said to be left ideal of *H* if *l*_1_ + *l*_2_ ∈ *L* for all *l*_1_, *l*_2_ ∈ *L*, and let *a* ∈ *H*, then ∃*l* ∈ *L* such that *al* ∈ *L*. The right ideals can be define dually.

In the case of a nonempty subset *N* of semiring *H*, the *h*-closure of *N* is defined by

(2) $$\begin{array}{c} \overset{¯}{N}=\left\{j\in H\;|\;j+n_{1}+i=n_{2}+i,\;\text{for some }n_{1},n_{2}\in N,i\in H\right\}. \end{array}$$

Since *H* is commutative, so *n* + *n* = *n* for all *n* ∈ *H*, $N\subseteq \overset{¯}{N.}$ Let $j\in \overset{¯}{N}$, then *j* + *n*_1_ + *i* = *n*_2_ + *i*, for some *n*_1_, *n*_2_ ∈ *N*, *i* ∈ *H*. Also, *j* + *j* + *n*_1_ + *i* = *j* + *n*_2_ + *i*⇒*j* + *n*_1_ + *i* = *j* + *n*_2_ + *i*⇒*n*_2_ + *i* = *j* + *n*_2_ + *i*. Since (*H*, +) is supposed to be idempotent, $\overset{¯}{N}=\left\{j\in H|j+n+i=n+i;\text{for some},n\in N,i\in H\right\}$ and $\overset{¯}{\overset{¯}{N}}=N$. *N* is called a *h*-set if $\overset{¯}{N}=N$.

A left ideal *N* of a semiring *H* is called a left *h*-ideal if for any *i* ∈ *H*, there exists *n*_1_, *n*_2_ ∈ *N* such that *i* + *n*_1_ + *j* = *n*_2_ + *j*, for *j* ∈ *H*.

A left (resp.right) ideal *N* of semiring *H* is a left (resp.right) *h*-ideal if it is *h*-set. We can say that, if *N* is the left *h*-ideal of *H*, then $\overset{¯}{N}$ is the smallest *h*-ideal of *H* containing *N*. We can also write $\overset{¯}{\overset{¯}{N}}=\overset{¯}{N}$ for every *N*⊆*H*. Further, $N\subseteq M\subseteq H\Rightarrow \overset{¯}{N}\subseteq \overset{¯}{M}$.

The intersection of left (resp. right) *h*-ideal is again *h*-ideal (if it is nonempty). There is the smallest left (resp. right) *h*-ideal that contains *n* ∈ *H*. This is called the left (resp. right) *h*-ideal generated by *n* and is denoted by *L*_*h*_(*n*)(resp.*R*_*h*_(*n*)).

**Definition 1 .**

Let *H* be a semiring and *N* be the subsemiring of *H*, then *N* is *h*-bi-ideal of *H* if *NHN*⊆*N* and $N=\overset{¯}{N}.$

A nonempty subset *N* of *H* is called a generalized *h*-bi-ideal of *H* if *NHN*⊆*N* and $N=\overset{¯}{N}.$

Let *u* ∈ *H*. We define *B*[*u*] ={{*x*_1_ + *x*_2_ + *x*_3_ ⋯ +*x*_*n*_} ∈ {*u*} ∪ {*u*^2^} ∪ *uHu*}. Then, *B*[*u*] be a subsemiring of semiring *H*. Further, ∀*h* ∈ *H* and *x*, *y* ∈ {*u*} ∪ {*u*^2^} ∪ *uHu*. We get *xhy* ∈ *Hu* which refers that *B*[*u*]*HB*[*u*]⊆*B*[*u*] and thus *B*[*u*] be a bi-ideal of *H*.

The article "Some Study of Semigroups of h-Bi-Ideals of Semirings" was retracted in 2023. Reasons: suspected computer-generated content; unreliable results or conclusions; concerns about the data; concerns about the results or conclusions.

**Lemma 1 .**

Let *H* be a semiring and let take *u* from *H*. Then, the principal *h*-bi-ideal of *H* generated by *u* is given by:

(3) $$\begin{array}{c} B_{h}\left(u\right)=\left\{v\in H\;|\;v+u+u^{2}+utu+w=u+u^{2}+utu+w,\text{for some }t\in H;w\in H\right\}. \end{array}$$

**Proof**

Let *x*, *y*∈*B*_*h*_(*u*). Then, ∃*m*, *n* ∈ *H* and *u* ∈ *H* such that *x* + *u* + *u*^2^ + *umu* + *w* = *u* + *u*^2^ + *umu* + *w* and *y* + *u* + *u*^2^ + *unu* + *w*′ = *u* + *u*^2^ + *unu* + *w*′ for *w* ∈ *H*. Then, we have:

(4) $$\begin{array}{c} x+u+u^{2}+umu+w=u+u^{2}+umu+w,\\ xy+\left(u+u^{2}+umu+w\right)y=\left(u+u^{2}+umu+w\right)y,\\ xy+\left(u+u^{2}+umu+w\right)\left(y+u+u^{2}+unu+w^{\prime }\right)=\left(u+u^{2}+umu+w\right)\left(y+u+u^{2}+unu+{\text{w}}^{\prime }\right),\\ xy+\left(u+u^{2}+umu+w\right)\left(u+u^{2}+unu+w^{\prime }\right)=\left(u+u^{2}+umu+w\right)\left(u+u^{2}+unu+w^{\prime }\right),\\ xy+u+u^{2}+uzu+{\text{w}}^{\prime \prime }=u+u^{2}+uzu+w^{\prime \prime }, \end{array}$$

since (*H*, +) is semillatice, where

(5) $$\begin{array}{c} z=u+u^{2}+un+mu+u^{2}n+mu^{2}+mu^{2}n+mw^{\prime }+wn\text{and}ww^{\prime }=w^{\prime \prime }, \end{array}$$

and so, *xy* ∈ *B*_*h*_(*u*). Also, *x* + *y* ∈ *B*_*h*_(*u*). Thus, *B*_*h*_(*u*) is a subsemiring of *H*. Similarly, *xmy* ∈ *B*_*h*_(*u*) for all *x*, *y* ∈ *B*_*h*_(*u*) and *m* ∈ *H*. Thus, *B*_*h*_(*u*) is a bi-ideal of *H*. Indeed $B_{h}\left(u\right)=\overset{¯}{B\left[u\right]},$ the *h*−closure of *B*[*u*]. Hence, *B*_*h*_(*u*) is a *h*-bi-ideal of *H*. Let *u* ∈ *B* and let *B* be a *h*-bi-ideal of semiring *H*. Let *x* ∈ *B*_*h*_(*u*), then there exists *m* ∈ *H* such that:

(6) $$\begin{array}{c} x+u+u^{2}+umu+w=u+u^{2}+umu+w\text{for}w\in H. \end{array}$$

Now, *u* ∈ *B* implies that *u* + *u*^2^ + *umu* + *w* ∈ *B* and so, *x* ∈ *B*. Hence, *B*_*h*_(*u*)⊆*B*. Thus, *B*_*h*_(*u*) is the least *h*-bi-ideal of *H*, which contains *u*.

**Theorem 1 .**

The set of all *h*-bi-ideals, the set of all left *h*-ideals, and the set of all right *h*-ideals shall be each semigroup with respect to the product of subsets of *H* specified in the usual way: ∗:*P*(*H*) × *P*(*H*)⟶*P*(*H*) by $M*N=\overset{¯}{MN.}$

**Proof**

Instead of defining binary operation on these three sets individually, we consider them to be semigroups of all subsets of *H*. Acknowledge receipt by *P*(*H*) of all subsets of *H*. We represent set of all *h*-bi-ideal by *B*(*H*), set of all left *h*-ideal by *ℒ*(*H*), and set of right *h*-ideal by *ℛ*(*H*). We define a binary operation ∗:*P*(*H*) × *P*(*H*)⟶*P*(*H*) by $M*N=\overset{¯}{MN}$.

The article "Some Study of Semigroups of h-Bi-Ideals of Semirings" was retracted in 2023. Reasons: suspected computer-generated content; unreliable results or conclusions; concerns about the data; concerns about the results or conclusions.

As *MN* = {*mn* | *m* ∈ *M*, *n* ∈ *N*}; so,

(7) $$\begin{array}{c} \overset{¯}{MN}=\left\{i\in H\;|\;i+m_{1}n_{1}+j=m_{2}n_{2}+j,m_{i}\in M,n_{i}\in N;i=1,2,..\text{and}j\in H\right\}. \end{array}$$

We will check that *P*(*H*) is a semigroup under the usual operation ∗. Also, since *L*_1_ and *L*_2_ are left *h*-ideal, then $\overset{¯}{L_{1}L_{2}}$ will become left *h*-ideal. So, ∗:*P*(*H*) × *P*(*H*)⟶*P*(*H*) induced a binary operation on *ℒ*(*H*); in the interests of comfort, we signify with the same symbol “∗.” Thus, *ℒ*(*H*) is a semigroup under the defined operation “∗.” Analogously, (*ℛ*(*H*) is a semigroup under the same binary operation “∗.” Now, we can show that the same holds for *B*(*H*).

Let *M* and *N* be the *h*-bi-ideals of semiring *H*. Let $u,v\in M*N=\overset{¯}{MN}$, then there exists *m* ∈ *M* and *n* ∈ *N* such that

(8) $$\begin{array}{c} u+mn+j=mn+j;v+mn+j^{\prime }=mn+j^{\prime };j,j^{\prime }\in H, \end{array}$$

then

(9) $$\begin{array}{c} u+v+mn+mn+j+j^{\prime }=mn+mn+j+j^{\prime },\\ u+v+mn+j^{\prime \prime }=mn+j^{\prime \prime }\&u+mn+j=mn+j, \end{array}$$

where *j* + *j*′ = *j*′′and *mn* + *mn* = *mn*. Since (*H*, +) is semillatice, so

(10) $$\begin{array}{c} \Rightarrow \left(u+mn+j\right)v=\left(mn+j\right)v,\\ \Rightarrow uv+\left(mn+j\right)v=\left(mn+j\right)v,\\ \Rightarrow uv+\left(mn+j\right)\left(v+mn+j^{\prime }\right)=\left(mn+j\right)\left(v+mn+j^{\prime }\right),\\ \Rightarrow uv+\left(mn+j\right)\left(mn+j^{\prime }\right)=\left(mn+j\right)\left(mn+j^{\prime }\right),\\ \Rightarrow uv+mnmn+mnj^{\prime }+jmn+jj^{\prime }=mnmn+mnj^{\prime }+jmn+jj^{\prime },\\ \Rightarrow uv+mnmn+j_{1}=mnmn+mnj+j_{1}, \end{array}$$

where *j*_1_ = *mnj*′ + *jmn* + *jj*′. ⇒*u* + *v* & *uv* both belong to $\overset{¯}{MN}.$ Also, for *h* ∈ *H*, we have *uhv* + *mnhmn* + *j*_1_*h* = *mnhmn* + *j*_1_*h* implies that $uhv\in \overset{¯}{MNHMN}\subseteq \overset{¯}{MN}\Rightarrow \overset{¯}{MN}H\overset{¯}{\text{M}N}\subseteq \overset{¯}{MN}.$ As $\overset{¯}{MN}$ is *h*-closure of *MN* & $\overset{¯}{MN}=MN$, i.e., *h*-subset of *H*. Thus, $\overset{¯}{MN}$ be *h*-bi-ideal of *H*. This shows that *B*(*H*) is a semigroup.

**Example 1 .**

Now, consider the semiring *S* = {0, *d*, *e*, *f*} defined by the following tables.

(11) $$\begin{array}{c} \begin{array}{ccccc} + & 0 & d & e & f\\ 0 & 0 & d & e & f\\ d & d & e & f & d\\ e & e & f & d & e\\ f & f & d & e & f \end{array}\;\begin{array}{ccccc} \cdot & 0 & d & e & f\\ 0 & 0 & 0 & 0 & 0\\ d & 0 & d & e & f\\ e & 0 & e & e & f\\ f & 0 & f & e & f \end{array} \end{array}$$

The only *h*-ideal is *S* itself. Obviously, this *h*-ideal is *h*-bi-ideal which forms a semigroup.

The article "Some Study of Semigroups of h-Bi-Ideals of Semirings" was retracted in 2023. Reasons: suspected computer-generated content; unreliable results or conclusions; concerns about the data; concerns about the results or conclusions.

## 3. Semigroup of *h*-Bi-Ideals in *h*-Regular Semirings

Suppose *H* be a semigroup, then *H* is said to be a regular semigroup if for each *t* ∈ *H*, there exists *u*′ ∈ *H* such that *t* = *tu*′*t*. Bourne [24] has described a semiring *S* to be regular if *u*′, *v*′ ∈ *H* exists for each *a* ∈ *H* that *t* + *tu*′*t* = *tv*′*t*. Adhikari [32] defined *k*-regularity; let *H* be a semiring, if (*H*, +) is a semillatice, then *t* + *tu*′*t* = *tv*′*t*. Adding *tu*′*t* + *tv*′*t* to both sides, that *t* + *t*(*u*′ + *v*′)*t* = *t*(*u*′ + *v*′)*t*. We can say that a semiring *H* ∈ *HL*^+^ is called *k*-regular if and only if for any *t* ∈ *H*, there is *u*′ ∈ *H* such that *t* + *tu*′*t* = *tu*′*t*.

**Definition 2 .**

A semiring *H* is called *h*-regular if ∀*t*′ ∈ *H*, then ∃*u*′, *v*′ ∈ *H* such that *t*′ + *t*′*u*′*t*′ + *w* = *t*′*v*′*t*′ + *w*, for *w* ∈ *H*.

Let *H* be a semiring, if (*H*, +) is a semillatice, then *t* + *tu*′*t*+*w* = *tv*′*t* + *w*. Adding *tu*′*t* + *tv*′*t* to both sides, then *t* + *t*(*u*′ + *v*′)*t* + *w* = *t*(*u*′ + *v*′)*t* + *w*. We can say that a semiring *H* ∈ *HL*^+^ is called *h*-regular if and only if for any *t* ∈ *H*, there is *u*′ ∈ *H* such that *t* + *tu*′*t* + *w* = *tu*′*t* + *w*.

**Theorem 2 .**

The following conditions are identical for the semiring *H*.

- *H* is *h*-regular
- For every *h*-bi-ideal *B* of *H*, $B=\overset{¯}{BHB}$
- For every generalized *h*-bi-ideal *M* of *H*, $M=\overset{¯}{MSM}$

**Proof**

(*iii*)⇒(*ii*) We know that every *h*-bi-ideal is a generalized *h*-bi-ideal from definition, so it is obvious.

(*i*)⇒(*iii*) Assume that *H* is *h*-regular and let *M* be the generalized *h*-bi-ideal of *H*. Then, *MHM*⊆*M* refers to $\overset{¯}{MHM}\subseteq \overset{¯}{M}H\overset{¯}{M}\subseteq \overset{¯}{M}\subseteq M$. Let *u* ∈ *M*, since *H* is *h*-regular, then there exists *m*′ ∈ *H* such that *u* + *um*′*u* + *w* = *um*′*u* + *w* for *w* ∈ *H*. Now, *um*′*u* ∈ *MHM* implies that $u\in \overset{¯}{MHM}$ and so $M\subseteq \overset{¯}{MHM}$. Thus, $M=\overset{¯}{MHM}$

(*ii*)⇒(*i*) Let *u*′ ∈ *H*, consider the *h*-bi-ideal *B*_*h*_(*u*′). Then, $u^{\prime }\in B_{h}\left(u^{\prime }\right)=\overset{¯}{B_{h}\left(u^{\prime }\right)HB_{h}\left(u^{\prime }\right)}$ implies that there exists *n*_1_, *n*_2_, *n*_3_, *n*_4_ ∈ *B*_*h*_(*u*′), and *h*_1_, *h*_2_ ∈ *H* such that

(12) $$\begin{array}{c} u^{\prime }+n_{1}h_{1}n_{2}+w=n_{3}h_{2}n_{4}+w,\text{for }w\in H,\\ \Rightarrow u^{\prime }+\left(n_{1}+n_{2}+n_{3}+n_{4}\right)\left(h_{1}+h_{2}\right)\left(n_{1}+n_{2}+n_{3}+n_{4}\right)+w=\left(n_{1}+n_{2}+n_{3}+n_{4}\right)\left(h_{1}+h_{2}\right)\left(n_{1}+n_{2}+n_{3}+n_{4}\right)+w,\\ \Rightarrow u^{\prime }+nhn+w=nhn+w, \end{array}$$

where *n* = *n*_1_ + *n*_2_ + *n*_3_ + *n*_4_ ∈ *B*_*h*_(*u*′) and *h* = *h*_1_ + *h*_2_ ∈ *H*. Hence, ∃*h* ∈ *H* such that

(13) $$\begin{array}{c} n+u^{\prime }+u^{\prime 2}+u^{\prime }hu^{\prime }+w=u^{\prime }+u^{\prime 2}+u^{\prime }hu^{\prime }+w, \end{array}$$

then we have

(14) $$\begin{array}{c} u^{\prime }+nhn+w=nhn+w\Rightarrow u^{\prime }+\left(n+u^{\prime }+u^{\prime 2}+u^{\prime }hu^{\prime }+w^{\prime }\right)h\left(n+u^{\prime }+u^{\prime 2}+u^{\prime }hu^{\prime }+w^{\prime }\right)+w=\left(n+u^{\prime }+u^{\prime 2}+u^{\prime }hu^{\prime }+w^{\prime }\right)h\left(n+u^{\prime }+u^{\prime 2}+u^{\prime }hu^{\prime }+w^{\prime }\right)+w\Rightarrow u^{\prime }+\left(u^{\prime }+u^{{\;}^{\prime }2}+u^{\prime }hu^{\prime }+w^{\prime }\right)h\left(u^{\prime }+u^{\prime 2}+u^{\prime }hu^{\prime }+w^{\prime }\right)+w\left(u^{\prime }+u^{\prime 2}+u^{\prime }hu^{\prime }+w^{\prime }\right)h\left(u^{\prime }+u^{\prime 2}+u^{\prime }hu^{\prime }+w^{\prime }\right)+w\Rightarrow u^{\prime }+u^{\prime }tu^{\prime }+w=u^{\prime }tu^{\prime }+w,\text{for some }t\in H, \end{array}$$

where *t* = *u*′ + *u*^′2^ + *u*′*h*^2^ + *u*^′2^*h*^2^ + *h*^3^*u*^′2^ + *h*^2^*w*′ + *w*′*h*^2^, and *w*′*w*′ = *w*. Thus, *H* is *h*-regular.

The article "Some Study of Semigroups of h-Bi-Ideals of Semirings" was retracted in 2023. Reasons: suspected computer-generated content; unreliable results or conclusions; concerns about the data; concerns about the results or conclusions.

**Lemma 2 .**

Subsemigroup *ℛ*(*H*) and (*ℒ*(*H*)) are bands for *h-*regular semiring *H*.

**Proof**

Let *ℛ*(*H*) and *ℒ*(*H*) are two subsemigroups. Let R′ ∈ *ℛ*(*H*) and *u* ∈ R′, then ∃*m* ∈ *H* such that *u* + *umu* + *w* = *umu* + *w* for *w* ∈ *H*. Now,

*um* ∈ *R*′*H*⊆*R*′ implies that $u\in R^{\prime 2}=\overset{¯}{R^{\prime }R^{\prime }}$, and so, *R*′⊆*R*^′2^. Also, it is obvious that *R*^′2^⊆*R*′. Thus, it can be written as *R*′ = *R*^′2^. Hence, *ℛ*(*H*) is a band.

Similarly, *ℒ*(*H*) is a band that can prove dually.

In the following theorem, we will prove that semigroup of all *h*-bi-ideals *B*(*H*) is a product of *ℛ*(*H*) and *ℒ*(*H*) semigroups. Bear in mind that *ℛ*(*H*)*ℒ*(*H*) = {*RL* | *R*′ ∈ *ℛ*(*H*), *L*′ ∈ *ℒ*(*H*)}.

**Theorem 3 .**

Show that *B*(*H*) = *ℛ*(*H*)*ℒ*(*H*) for *h*-regular semiring *H*.

**Proof**

To prove that *B*(*H*) = *ℛ*(*H*)*ℒ*(*H*), we have to show that *B*(*H*)⊆*ℛ*(*H*)*ℒ*(*H*) and *ℛ*(*H*)*ℒ*(*H*)⊆*B*(*H*). Suppose *R*′ ∈ *ℛ*(*H*) and *L*′ ∈ *ℒ*(*H*) and we represent $B=R^{\prime }*L^{\prime }=\overset{¯}{R^{\prime }L^{\prime }}$. So, *B* is *h*-subsemiring of *H*. Now, $BHB=\overset{¯}{R^{\prime }L^{\prime }}H\overset{¯}{R^{\prime }L^{\prime }}\subseteq \overset{¯}{R^{\prime }L^{\prime }HR^{\prime }L^{\prime }}\subseteq \overset{¯}{R^{\prime }L^{\prime }}=B$. This shows *B* ∈ *B*(*H*). Hence, *ℛ*(*H*)*ℒ*(*H*)⊆*B*(*H*).

Now, suppose *B* ∈ *B*(*H*). We represent $L^{\prime }=\overset{¯}{HBUB}$ and $R^{\prime }=\overset{¯}{BHUB}.$ Then, $HL=H\overset{¯}{HBUB}$$\subseteq \overset{¯}{HHBUB}=\overset{¯}{HB}\subseteq \overset{¯}{HBUB}=L^{\prime }$ refers that *L*′ is left *h*-ideal of *H*. Now, $R^{\prime }H=\overset{¯}{BHUB}H\subseteq \overset{¯}{BHUBH}=\overset{¯}{BH}\subseteq \overset{¯}{BHUB}=R^{\prime }$ implies that *R*′ is right *h*-ideal of *H*. Now, $\overset{¯}{R^{\prime }L^{\prime }}=\overset{¯}{\overset{¯}{BHUB}\overset{¯}{HBUB}}\subseteq \overset{¯}{\left(BHUB\right)\left(HBUB\right)}\subseteq \overset{¯}{BHBUB^{2}}\subseteq \overset{¯}{B}=B$. Also, $B\subseteq HBUB\subseteq \overset{¯}{HBUB}=L^{\prime }$ and $B\subseteq BHUB\subseteq \overset{¯}{BHUB}=R^{\prime }$. Since *H* is *h*-regular, and we know that *H* is *h*-regular iff$B=\overset{¯}{BHB}$ for every *h*-bi-ideal *B* of *H*. So, $B=\overset{¯}{BHB}$ implies that $B\subseteq \overset{¯}{R^{\prime }HL^{\prime }}\subseteq \overset{¯}{R^{\prime }L^{\prime }}.$ Hence, $B=\overset{¯}{R^{\prime }L^{\prime }}$ and so *B*(*H*)⊆*ℛ*(*H*)*ℒ*(*H*). Thus, *B*(*H*) = *ℛ*(*H*)*ℒ*(*H*). Hence, proved.

The article "Some Study of Semigroups of h-Bi-Ideals of Semirings" was retracted in 2023. Reasons: suspected computer-generated content; unreliable results or conclusions; concerns about the data; concerns about the results or conclusions.

## 4. Semigroup of *h*-Bi-Ideals in *h*-Clifford and Left *h*-Clifford Semiring

In this segment, we are characterizing the semigroup of all *h*-bi-ideals of the *h*-Clifford semiring and the left *h*-Clifford semiring.

**Definition 3 .**

Let *H* be a semiring, then *H* is called a *h-*Clifford semiring if

- *H* be a *h*-regular semiring, i.e., for every *t* ∈ *H*, then ∃*u*, *v* ∈ *H* such that *t* + *tut* + *w* = *tvt* + *w*; for *h* ∈ *H*
- $\overset{¯}{Ht}=\overset{¯}{tH}$ for every *t* ∈ *H*

**Definition 4 .**

An element *e* of semiring *H* is *h-*idempotent of *H* if *e* + *e*^2^ + *w* = *e*^2^ + *w* for *w* ∈ *H*. *E*_*h*_(*H*) is representation of set of all *h-*idempotents.

**Theorem 4 .**

In *h*-regular semiring (*H*, +, ·), the given following statements are identical

- *H* be *h*-Clifford semiring

(15) $$\begin{array}{c} \overset{¯}{L}=\overset{¯}{R}, \end{array}$$

(ii) $\overset{¯}{uH}=\overset{¯}{Hu}$ for all *u* ∈ *H*
(iii) All left *h*-ideals as well as all right *h*-ideals are two sided and $T_{1}\cap T_{2}=\overset{¯}{T_{2}T_{1}}$ for any two of them
(iv) $L\cap R=\overset{¯}{LR}$ for all left *h*-ideal and for all right *h*-ideals *R*
(v) $L_{1}\cap L_{2}=\overset{¯}{L_{1}L_{2}}$ for any two left *h*-ideals *L*_1_, *L*_2_ of *H* and $R_{1}\cap R_{2}=\overset{¯}{R_{1}R_{2}}$ for any two right *h*-ideals *R*_1_, *R*_2_ of *H*

**Proof**

(*i*)⇒(*ii*) Suppose *H* is *h*-Clifford and we want to show that $\overset{¯}{ℒ}=\overset{¯}{ℛ}.$ For this, we have to prove that $\overset{¯}{ℒ}$ and $\overset{¯}{ℛ}$ are subsets of each other. For this, let $\left(u,v\right)\in \overset{¯}{ℒ}$ for *u*, *v* ∈ *H*, then ∃*t* ∈ *H* such that

(16) $$\begin{array}{c} u+tv+w=tv+w,\text{for }w\in H, \end{array}$$

(17) $$\begin{array}{c} v+tu+w^{\prime }=tu+w^{\prime },\text{for }w^{\prime }\in H, \end{array}$$

since *H* is *h*-regular, then there is *h*_1_, *h*_2_ ∈ *H* such that *u* + u*h*_1_*u* + *w* = *uh*_1_*u* + *w* and *v* + *vh*_2_*v* + *w*′ = *vh*_2_*v* + *w*′. Now, *u* + *uh*_1_*u* + *uh*_1_*tv* + *w* + *w*′ = *uh*_1_*u* + *uh*_1_*tv* + *w* + *w*′; this implies that *u* + *uh*_1_*u* + *uh*_1_*tv* + *w* = *uh*_1_*u* + *uh*_1_*tv* + *w*, where *w* + *w*′ = *w*. Hence, by (16), *u* + *uh*_1_*tv* + *w* = *uh*_1_*tv* + *w*. Similarly, *v* + *vh*_2_*tu* + *w*′ = *vh*_2_*tu* + *w*′. Since (*H*, +) is a semillatice, these implies that

(18) $$\begin{array}{c} u+uxu+w=uxu+w, \end{array}$$

(19) $$\begin{array}{c} v+vxv+w^{\prime }=vxv+w^{\prime }, \end{array}$$

(20) $$\begin{array}{c} u+uxv+w=uxv+w, \end{array}$$

(21) $$\begin{array}{c} v+vxu+w^{\prime }=vxu+w^{\prime }, \end{array}$$

where *x* = *h*_1_ + *h*_2_ + *h*_1_*t* + *h*_2_*t*. Thus, *ux* and *vx* are *h*-idempotents. Since *H* is a *h*-Clifford semiring, there are *s*_1_, *s*_2_ in *H* such that *u* + *vs*_1_*v* + *w* = *vs*_1_*v* + *w* and *vxu* + *us*_2_*u* + *w*′′ = *us*_2_*u* + *w*′′for *w*′′ ∈ *H*. Hence, (20) and (21) refers that *u* + *vs*_1_*v* + *w* = *vs*_1_*v* + *w* and *v* + *us*_2_*u* + *w*′ = *us*_2_*u* + *w*′. Therefore, $u\overset{¯}{ℛ}v.$ Hence, $\overset{¯}{ℒ}\subseteq \overset{¯}{ℛ}$. Similarly, $\overset{¯}{ℛ}\subseteq \overset{¯}{ℒ}.$ Thus, $\overset{¯}{ℒ}=\overset{¯}{ℛ}.$

(*ii*)⇒(*iii*) Suppose that $\overset{¯}{ℒ}=\overset{¯}{ℛ}$. We will prove that $\overset{¯}{uH}=\overset{¯}{Hu}$ for all *u* ∈ *H*. For this, let $v\in \overset{¯}{uH}$, then there is *t*_1_ ∈ *H* such that *v* + *ut*_1_ + *w*′ = *ut*_1_ + *w*′ for *w*′ ∈ *H*. Since *H* is *h*-regular, there is *t*_2_ ∈ *H* for which *u* + *ut*_2_*u* + *w* = *ut*_2_*u* + *w*. Thus, there is *t* = *t*_1_ + *t*_2_ ∈ *H* such that *v* + *ut* + *w*′ = *ut* + *w*′ and *u* + *utu* + *w* = *utu* + *w*. This implies that $u\overset{¯}{ℛ}ut,$ so $ut\overset{¯}{ℒ}u$. Therefore, there is *x* ∈ *H* such that *ut* + *xu* + *w* = *xu* + *w*. Now, *v* + *ut* + *xu* + *w*′ = *ut* + *xu* + *w*′ implies that *v* + *xu* + *w*′ = *xu* + *w*′, that is, $v\in \overset{¯}{Hu}.$ Thus, $\overset{¯}{uH}\subseteq \overset{¯}{Hu}$. Similarly, $\overset{¯}{Hu}\subseteq \overset{¯}{uH}$. Therefore, $\overset{¯}{uH}=\overset{¯}{Hu}$.

(*iii*)⇒(*iv*) Lets take *u* from left *h*-ideal *L*, and *t* ∈ *H*, then $ut\in \overset{¯}{uH}=\overset{¯}{Hu}\subseteq L$ implies that *L* is two-sided *h*-ideal. Similarly, this will be hold for right *h*-ideal *R*. Let *M* and *N* are two *h*-ideals of *H*. Then, *MN* contain in *M*∩*N*. Let *u* ∈ *M*∩*N*, since *H* is *h*-regular, there is *h* ∈ *H* such that *u* + *utu* + *w* = *utu* + *w* for *w* ∈ *H*. So, *u* will be in $\overset{¯}{MN}$, thus $M\cap N\subseteq \overset{¯}{MN}$. Therefore, $M\cap N\subseteq \overset{¯}{MN}$.

(*iv*)⇒(*v*) This is trivial.

(*v*)⇒(*i*) Let *u* ∈ *H* and *e* be *h*-idempotent in *H*. Then, from (*v*), we can write $\overset{¯}{\overset{¯}{Hu}.\overset{¯}{eH}}=\overset{¯}{Hu}\cap \overset{¯}{eH}$. Since *H* is *h*-regular, there is *t* ∈ *H* such that *ue* + *uetue* + *w*_1_ = *uetue* + *w*_1_ for *w*_1_ ∈ *H* and so,

(22) $$\begin{array}{c} ue+uetuetue+w_{1}=uetuetue+w_{1}. \end{array}$$

Now, *ue* + ((*uet*)*u*)(*e*(*tue*)) + *w*_1_ = ((*uet*)*u*)(*e*(*tue*)) + *w*_1_ implies that $ue\in \overset{¯}{\overset{¯}{Hu}.\overset{¯}{eH}}$ and so, $ue\in \overset{¯}{Hu}.$ Hence, there is *p* ∈ *H* such that *ue* + *pu* + *w*_2_ = *pu* + *w*_2_. Now, (22) implies that

(23) $$\begin{array}{c} ue+uetuet\left(ue+pu+w_{2}\right)+w_{1}=uetuet\left(ue+pu+w_{2}\right)+w_{1}, \end{array}$$

that is,

(24) $$\begin{array}{c} ue+u\left(etuetp\right)u+uetuetw_{2}+w_{1}=u\left(etuetp\right)u+uetuetw_{2}+w_{1}. \end{array}$$

Thus, *ue* + *us*_1_*u* + *w*_3_ = *us*_1_*u* + *w*_3_, where *s*_1_ = *etuetp* and *uetuetw*_2_ + *w*_1_ = *w*_3_. Similarly, there is *s*_2_ ∈ *H* such that *eu* + *us*_2_*u* + *w*_4_ = *us*_2_*u* + *w*_4_. Therefore, *ue* + *usu* + *w* = *usu* = *w* and *eu* + *usu* + *w* = *usu* + *w*, where *s* = *s*_1_ + *s*_2_ and *w*_3_ + *w*_4_ = *w*. Hence, *H* is *h*-Clifford.

(*iv*)⇒(*vi*) This is trivial.

(*vi*)⇒(*i*) Let *u* ∈ *H* and *e* ∈ *E*_*h*_(*H*). Since *H* is *h*-regular semiring, there is *t* ∈ *H* such that *ue* + *uetue* + *w*_5_ = *uetue* + *w*_5_ for *w*_5_ ∈ *H*, and so,

(25) $$\begin{array}{c} ue+uetuetue+w_{5}=uetuetue+w_{5}. \end{array}$$

Now, *ue* + (*uet*)*u*(*etu*)*e* + *w* = (*uet*)*u*(*etu*)*e* + *w* implies that $ue\in \overset{¯}{\overset{¯}{Hu}.\overset{¯}{He}}=\overset{¯}{Hu}\cap \overset{¯}{He}$. Then, $ue\in \overset{¯}{Hu}$ implies that there is *p* ∈ *H* such that *ue* + *pu* + *w*_6_ = *pu* + *w*_6_. Hence, (25) implies that

(26) $$\begin{array}{c} ue+uetuet\left(ue+pu+w_{6}\right)+w_{5}=uetuet\left(ue+pu+w_{6}\right)+w_{5}, \end{array}$$

that is,

(27) $$\begin{array}{c} ue+u\left(etuetp\right)u+uetuetw_{6}+w_{5}=u\left(etuetp\right)u+uetuetw_{6}+w_{5}. \end{array}$$

Thus, *ue* + *us*_3_*u* + *w*_7_ = *us*_3_*u* + *w*_7_, where *s*_3_ = *etuetp* and *uetuetw*_6_ + *w*_5_ = *w*_7_. Similarly, there is *s*_2_ ∈ *H* such that *eu* + *us*_4_ + *w*_8_ = *us*_4_ + *w*_8_. Therefore, *ue* + *usu* + *w* = *usu* + *w* and *eu* + *usu* + *w* = *usu* + *w*, where *s*_3_ + *s*_4_ = *s* and *w*_7_ + *w*_8_ = *w*. Hence, *H* is *h*-Clifford.

The article "Some Study of Semigroups of h-Bi-Ideals of Semirings" was retracted in 2023. Reasons: suspected computer-generated content; unreliable results or conclusions; concerns about the data; concerns about the results or conclusions.

**Theorem 5 .**

Let *H* be *h-*regular semiring. Then, *H* is *h-*Clifford if and only if for all *u*, *v* ∈ *H*, there is *t* ∈ *H* such that

(28) $$\begin{array}{c} uv+utu+w_{1}=utu+w_{1},\text{for }w_{1}\in H,\\ vu+utu+w_{2}=utu+w_{2},\text{for }w_{2}\in H. \end{array}$$

**Proof**

Let *H* be a semiring, and for all *u*, *v* ∈ *H*, there is *t* ∈ *H* such that

(29) $$\begin{array}{c} uv+utu+w_{1}=utu+w_{1}, \end{array}$$

(30) $$\begin{array}{c} vu+utu+w_{2}=utu+w_{2}. \end{array}$$

Let *u* ∈ *H* and $m\in \overset{¯}{uH}$. Then, there is *x* ∈ *H* such that *m* + *ux* + *w*_3_ = *ux* + *w*_3_ for *w*_3_ ∈ *H*. Now, (29) implies that *ux* + *utu* + *w*_1_ = *utu* + *w*_1_ for some *t* ∈ *H*. Therefore, *m* + *utu* + *w*_1_ = *utu* + *w*_1_. Hence, $m\in \overset{¯}{Hu}$. Thus, $\overset{¯}{uH}\subseteq \overset{¯}{Hu}$. Similarly, $\overset{¯}{Hu}\subseteq \overset{¯}{uH}$. Therefore, $\overset{¯}{uH}=\overset{¯}{Hu}$. Hence, *H* is *h*-Clifford.

Conversely, let *H* be *h*-Clifford and *u*, *v* ∈ *H*. Since *H* is *h*-regular, there is *t* ∈ *H* such that

(31) $$\begin{array}{c} uv+uvtuv+w_{1}=uvtuv+w_{1},\text{for }w\in H. \end{array}$$

Now, $uv\in \overset{¯}{uH}=\overset{¯}{Hu}$ implies that for some *x* ∈ *H*, *uv* + *xu* + *w*_1_ = *xu* + *w*_1_. Now, (31) implies that

(32) $$\begin{array}{c} uv+uvt\left(uv+xu+w_{1}\right)+w_{4}=uvt\left(uv+xu+w_{1}\right)+w_{4},\text{for }w_{4}\in H, \end{array}$$

and this implies that

(33) $$\begin{array}{c} uv+u\left(vtx\right)u+uvtw_{1}+w_{4}=u\left(vtx\right)u+uvtw_{1}+w_{4}. \end{array}$$

Thus, *s*_1_ = *vtx* ∈ *H* and *uvtw*_1_ + *w*_4_ = *w*_5_ ∈ *H* such that *uv* + *us*_1_*u* + *w*_5_ = *us*_1_*u* + *w*_5_. Similarly, there is *s*_2_ ∈ *H* such that *v* + *us*_2_*u* + w_6_ = *us*_2_ + *w*_6_, and then, *uv* + *usu* + *w* = *usu* + *w* and *vu* + *usu* + *w* = *usu* + *w*, where *s* = *s*_1_ + *s*_2_ and *w*_5_ + *w*_6_ = *w* ∈ *H*.

**Theorem 6 .**

Let *H* be *h-*regular semiring. Then, *H* is *h-*Clifford if and only if for all u, *v* ∈ *H*, there is *n* ∈ *H* such that

(34) $$\begin{array}{c} uv+vnu+w=vnu+w,\text{for }w\in H. \end{array}$$

**Proof**

Suppose that *H* be *h*-Clifford and let ∀*u*, *v* ∈ *H*. Since *H* is a *h*-regular, there exist *t* ∈ *H* such that

(35) $$\begin{array}{c} uv+uvt\text{u}v+w_{1}=uvtuv+w_{1},\text{for }w_{1}\in H. \end{array}$$

Now, $uv\in \overset{¯}{uH}=\overset{¯}{Hu}$, then there is *x*_1_ ∈ *H*, such that *uv* + *x*_1_*u* + *w*_2_ = *x*_1_*u* + *w*_2_, for *w*_2_ ∈ *H*. Similarly, $uv\in \overset{¯}{Hv}=\overset{¯}{vH}$; there is *x*_2_ ∈ *H*, such that *uv* + *vx*_2_ + *w*_3_ = *vx*_2_ + *w*_3_, for *w*_3_ ∈ *H*. Then, *uv* + *vnu* + *w* = *vnu* + *w*, for *w* ∈ *H* implies that

(36) $$\begin{array}{c} uv+\left(uv+vx_{2}+w_{3}\right)t\left(uv+x_{1}u+w_{2}\right)+w=\left(uv+vx_{2}+w_{3}\right)t\left(uv+x_{1}u+w_{2}\right)+w, \end{array}$$

or

(37) $$\begin{array}{c} uv+vx_{2}tx_{1}u+w_{3}tw_{3}+w=vx_{2}tx_{1}u+w_{3}tw_{3}+w. \end{array}$$

Hence, there is *n* = *x*_2_*tx*_1_ ∈ *H* and *w* = *w*_3_*tw*_3_ + *w* ∈ *H* such that *uv* + *vnu* + *w* = *vnu* + *w*.

Conversely, let *u* ∈ *H* and $t\in \overset{¯}{uH}$. Then, there exists *v* ∈ *H* such that *t* + *uv* + *w* = *uv* + *w*; *w* ∈ *H*. By our hypothesis, there is *n* ∈ *H* for which *uv* + *vnu* + *w* = *vnu* + *w*. Therefore, *t* + *vnu* + *w* = *vnu* + *w*. So, $t\in \overset{¯}{Hu}$. Thus, $\overset{¯}{Hu}$$\subseteq \overset{¯}{uH}$. Similarly, $\overset{¯}{uH}\subseteq \overset{¯}{Hu}.$ Therefore, $\overset{¯}{uH}=\overset{¯}{Hu}$. Hence, *H* is *h*-Clifford.

**Theorem 7 .**

In *h*-Clifford semiring *H* every *h-bi-*ideal is an *h*-ideal of *H*.

**Proof**

Suppose that *H* be *h*-Clifford semiring and let *B* ∈ *H* and we are to prove that *B* is *h*-bi-ideal of *H*. For this, let *m* ∈ *B* and *u* ∈ *H*. Then, ∃*x*, *y* ∈ *H* such that

(38) $$\begin{array}{c} um+mxm+w=mxm+w,\text{for }w\in H,\\ mu+mym+w=mym+w. \end{array}$$

Thus, $um,mu\in \overset{¯}{BHB}\subseteq \overset{¯}{B}=B$ which shows that *B* is *h*-ideal of $\dot{H}$. Hence, proved.

**Theorem 8 .**

Let *H* be semiring if semigroup of all *h-bi-*ideals (*B*(*H*), ∗) is semilattice, then prove that *H* is *h*-Clifford.

**Proof**

Assume that *B*(*H*) is semillatice, then *H* is *h*-regular semiring. Let *u*, *v* ∈ *H*, then *uv* ∈ *B*_*h*_(*u*)*B*_*h*_(*v*) = *B*_*h*_(*v*)*B*_*h*_(*u*) implies that *uv* + *rs* + *w* = *rs* + *w* for some *r* ∈ *B*_*h*_(*v*) and *s* ∈ *B*_*h*_(*u*) and for *w* ∈ *H*; since *H* is *h*-regular, there are *x*, *y* ∈ *H* such that *r* + v*xv* + *w*′ = *vxv* + *w*′ and *s* + *uyu* + *w*′′ = *uyu* + *w*′′ for *w*′, *w*′′ ∈ *H*. Then, we have *uv* + *rs* + *w* = *rs* + *w*

(39) $$\begin{array}{c} \Rightarrow uv+\left(r+vxv+w^{\prime }\right)\left(s+uyu+w^{\prime \prime }\right)+w=\left(r+vxv+w^{\prime }\right)\left(s+uyu+w^{\prime \prime }\right)+w,\\ \Rightarrow uv+v\left(xvuy\right)u+vxvw^{\prime }+w^{\prime }uyu+w^{\prime w^{\prime \prime }}=v\left(xvuy\right)u+vxvw^{\prime }+w^{\prime }uyu+w^{\prime }w^{\prime \prime },\\ \Rightarrow \text{uv}+\text{v}zu+w^{\prime \prime \prime }=vzu+w^{\prime \prime \prime }, \end{array}$$

where *z* = *xvuy* and *w*′′′ = *vxvw*′ + *w*′*uyu* + *w*′*w*′′ ∈ *H*.

Hence, *H* is a *h*-Clifford semiring.

**Theorem 9 .**

The set of all *h*-bi-ideals *B*(*H*) is a left normal band if and only if semiring is a left *h-*Clifford.

**Proof**

Let *H* be *h*-Clifford semiring. Let *L*, *M*, *N* ∈ *B*(*H*) and $t\in L*M*N=\overset{¯}{LMN}$. Then, for some *l* ∈ *L*, *m* ∈ *M*, and *n* ∈ *N*, we have *t* + *lmn* + *w* = *lmn* + *w* for *w* ∈ *H*. Since *H* is *h*-regular; there is *s* ∈ *H* such that *lmn* + *lmnslmn* + *w*_1_ = *lmnslmn* + *w*_1_ for *w*_1_ ∈ *H*, which implies that *t* + *lmnslmn* + *w* = *lmnslmn* + *w*, from which we get *t* + *lxlmnxnsls*_1_*n* + *w* = *lxlmnxnsls*_1_*n* + *w* as *l* + *lxl* + *w*′ = *lxl* + *w*′, *n* + *nxn* + *w*′′ = *nxn* + *w*′′, and *mn* + *s*_1_*m* + *w*′′′ = *s*_1_*m* + *w*′′′ for some *x*, *s*_1_ ∈ *H* and *w*′, *w*′′, *w*′′′ ∈ *H*. Again, since *lm* + *s*_2_*l* + *w*_1_ = *s*_2_*l* + *w*_1_ and *nsls*_1_ + *s*_3_*n* + *w*_2_ = *s*_3_*n* + *w*_2_; for some *s*_2_, *s*_3_ ∈ *H* and *w*_1_, *w*_2_ ∈ *H*, after rearranging the above expression, we get *t* + (*lxs*_2_*l*)(*nxs*_3_*n*)*m* + *w* = (l*xs*_2_*l*)(*nxs*_3_*n*)*m* + *w*. Thus, $t\in \overset{¯}{LMN}=L*M*N$. Therefore, *L*∗*M*∗*N*⊆*L*∗*N*∗*M*; similarly, it can be proved that *L*∗*N*∗*M* is subset of *L*∗*M*∗*N*. Hence, *L*∗*M*∗*N* = *L*∗*N*∗*M*, and so, *B*(*H*) is a left normal band.

Conversely, suppose that set of all *h*-bi-ideals *B*(*H*) be a left normal band and we are to prove that *H* is a left *h*-Clifford. Thus, *H* is *h*-regular, we know that semigroup *B*(*H*) is regular under ∗ iff *H* is *h*-regular. Using this result, let *u*, *v* ∈ *H*, then there is *t* ∈ *H* such that *uv* + *uvtuv* + *w* = *uvtuv* + *w* which implies that $uv\in \overset{¯}{B_{h}\left(uvt\right)B_{h}\left(u\right)B_{h}\left(v\right)}=\overset{¯}{B_{h}\left(uvt\right)B_{h}\left(v\right)B_{h}\left(u\right)}$; since *B*(*H*) is a left normal band, then *uv* + *opq* + *w*′ = *opq* + *w*′, where *o* ∈ *B*_*h*_(*uvt*), *p* ∈ *B*_*h*_(*v*), *q* ∈ *B*_*h*_(*u*), and *w*′ ∈ *H*. Since *H* is *h*-regular, there is *h* ∈ *H* such that *q* + *uhu* + *w*′′ = *uhu* + *w*′′. Now, *uv* + *opq* + *w*′ = *opq* + *w*′ implies that *uv* + (*opuh*)*u* + *w*′′′ = (*opuh*)*u* + *w*′′′, for *w*′′′ ∈ *H*. Thus, *H* is left *h*-Clifford.

The article "Some Study of Semigroups of h-Bi-Ideals of Semirings" was retracted in 2023. Reasons: suspected computer-generated content; unreliable results or conclusions; concerns about the data; concerns about the results or conclusions.

## 5. Semigroup of Minimal *h*-Bi-Ideals

We will define semiring in terms of minimal *h*-ideals in this section and will work on semiring of minimal left *h*-ideals and minimal right *h*-ideals. Also, we will look at those semirings *H* ∈ *HL*^+^ that have a minimal left(right)*h*-ideal, and a minimal *h*-bi-ideal. *B*_*m*_(*H*) stands for the class of all minimal *h*-bi-ideals. Likewise, we will denote minimal left and minimal right *h*-ideals with *ℒ*_*m*_(*H*) and *ℛ*_*m*_(*H*).

**Definition 5 .**

Let *H* be a semiring and *N* be the *h-bi-*ideal of *H*, then *N* be a minimal *h-*bi-ideal if for every nontrivial *h*-bi-ideal *U* of *H*, *U*⊆*N* follows that *U* = *N*.

**Theorem 10 .**

Let ∅≠*N*⊆*H* is a minimal *h*-bi-ideal of *H* if and only if $N\subseteq \overset{¯}{R_{1}L_{1}}$ and $\overset{¯}{R_{1}L_{1}}\subseteq N$ for minimal right and left *h*-ideal *R*_1_, *L*_1_ of *H*, respectively.

**Proof**

Let ∅≠*N*⊆*H*, suppose that *N* is a minimal *h*-bi-ideal of *H*, then $R_{1}=\overset{¯}{NH}$ and $L_{1}=\overset{¯}{HN}$ follows directly right *h*-ideal and left *h*-ideal, respectively. Let us take *R*_2_⊆*R*_1_ is a right *h*-ideal of *H*, then $\overset{¯}{R_{2}L}$ will be *h*-bi-ideal of *H*, this follows that $\overset{¯}{R_{2}L_{1}}\subseteq \overset{¯}{R_{1}L_{1}}\subseteq \overset{¯}{\overset{¯}{NH}\overset{¯}{HN}}\subseteq \overset{¯}{NHN}\subseteq \overset{¯}{N}H\overset{¯}{N}\subseteq \overset{¯}{N}=N$, by definition of minimality of *N*; $N=\overset{¯}{R_{2}L_{1}}$. This implies that $R_{1}=\overset{¯}{NH}=\overset{¯}{\overset{¯}{R_{2}L_{1}}H}\subseteq \overset{¯}{R_{2}H}\subseteq R_{2}$, and so, *R*_2_ = *R*_1_. Thus, $R_{1}=\overset{¯}{NH}$ will be a minimal right *h*-ideal of *H*. Likewise, $L_{1}=\overset{¯}{HN}$ is a minimal left *h*-ideal of *H*, since $\overset{¯}{R_{1}L_{1}}\subseteq N$ be a *h*-bi-ideal and *N* is a minimal *h*-b-ideal of $\dot{H}.$ Finally, $N=\overset{¯}{R_{1}L_{1}}.$ Hence, proved.

**Theorem 11 .**

If *B*_*m*_(*H*) is set of all minimal *h*-bi-ideals, then *B*_*m*_(*H*) is a subsemigroup of *B*(*H*).

**Proof**

Suppose two minimal *h*-bi-ideal *M*_1_and *M*_2_ in *B*_*m*_(*H*). Let *G* ∈ *B*(*H*) be such that $G\subseteq \overset{¯}{M_{1}M_{2}}$ then $\overset{¯}{GM_{1}},$$\overset{¯}{M_{2}G}\in B\left(H\right)$. Now, $\overset{¯}{GM_{1}}\subseteq M_{1}M_{2}M_{1}\subseteq M_{1}GM_{2}\subseteq M_{1}.$ Then, by minimality of *M*_1_, we have $\overset{¯}{GM_{1}}=M_{1}$. Similarly, $\overset{¯}{M_{2}G}=M_{2}.$Then, $\overset{¯}{M_{1}M_{2}}=\overset{¯}{\overset{¯}{GM_{1}}\overset{¯}{M_{2}G}}\subseteq \overset{¯}{GM_{1}M_{2}G}\subseteq \overset{¯}{GHG}\subseteq \overset{¯}{G}=G$. Therefore, $G=\overset{¯}{M_{1}M_{2}}$. Hence, the set *B*_*m*_(*H*) would be subsemigroup of *B*(*H*).

As the same pattern, the set *ℒ*_*m*_(*H*) and *ℛ*_*m*_(*H*) are subsemigroup of *B*(*H*) which can justify easily.

**Theorem 12 .**

(a) If a nonempty class of all minimal left *h*-ideals is *ℒ*_*m*_(*H*) and *L*_1_∈*ℒ*(*H*), then *L*_1_∗*L*_*m*_′ = *L*_*m*_′, where *L*_*m*_′ is in *ℒ*_*m*_(*H*). Hence, *ℒ*_*m*_(*H*) be a left ideal of semigroup, i.e., (*ℒ*(*H*), ∗), in particular a subsemigroup. Further, (*ℒ*_*m*_(*H*), ∗) be a right zero band.

(b) If a nonempty class of all minimal right *h*-ideals is *ℛ*_*m*_(*H*) and *R*_1_∈*ℛ*(*H*), then *R*_1_∗*R*_*m*_′ = *R*_*m*_′, where *R*_*m*_′ is in *ℛ*_*m*_(*H*). Hence, *ℛ*_*m*_(*H*) be a right ideal of semigroup, i.e., (*ℛ*(*H*), ∗), in particular, a subsemigroup. Further, (*ℛ*_*m*_(*H*), ∗) be a left zero band.

**Proof**

(a) For some *L*_1_ ∈ *ℒ*(*H*) and *L*_*m*_′∈*ℒ*_*m*_(*H*), take the left *h*-ideal *L*_1_∗*L*_*m*_′. Then, *L*_1_∗*L*_*m*_′ implies $L_{1}*L_{m}^{\prime }=\overset{¯}{L_{1}L_{m}^{\prime }}$, and this follows $\overset{¯}{L_{1}L_{m}^{\prime }}$$\subseteq \overset{¯}{L_{m}^{\prime }}$ = *L*_*m*_′ and by minimality of *L*_*m*_′ shows *L*_1_∗*L*_*m*_′ = *L*_*m*_′.

(b) This proceeds dually.

The article "Some Study of Semigroups of h-Bi-Ideals of Semirings" was retracted in 2023. Reasons: suspected computer-generated content; unreliable results or conclusions; concerns about the data; concerns about the results or conclusions.

**Theorem 13 .**

If set of all minimal *h*-bi-ideal *B*_*m*_(*H*) for a semiring *H* is nonempty, then ∀*M*_*m*_, *G*_*m*_ ∈ *B*_*m*_(*H*), and *B* ∈ *B*(*H*); there are *M*_*m*_∗*B*∗*G*_*m*_ ∈ *B*_*m*_(*H*), *M*_*m*_∗*M*_*m*_ = *M*_*m*_, and *M*_*m*_∗*B*∗*M*_*m*_ = *M*_*m*_. As a consequence, semigroup's bi-ideal is the set of all minimal *h*-bi-ideals (*B*_*m*_(*H*), ∗), in particular, a subsemigroup. Further, (*B*_*m*_(*H*), ∗) is rectangular band.

**Proof**

Let *B*_*m*_(*H*) is set of all minimal *h*-bi-ideal and *B*(*H*) denotes the set of *h*-bi-ideal, then suppose M_*m*_, *G*_*m*_ ∈ *B*_*m*_(*H*) and *B* ∈ *B*(*H*). Denote the bi-ideal *M*_*m*_∗*B*∗*G*_*m*_ by *G*. Let *F* ∈ *B*(*H*) such that *F*⊆*G*, then $F*M_{m}\subseteq \overset{¯}{M_{m}BG_{m}M_{m}}\subseteq M_{m}$, and minimality of *M*_*m*_ shows that *M*_*m*_ = *F*∗*M*_*m*_. Similarly, *G*_*m*_ = *G*_*m*_∗*F*; therefore, $G=M_{m}*B*G_{m}=F*M_{m}*B*G_{m}*F=\overset{¯}{FM_{m}BG_{m}F}\subseteq F$, and so, *G* = *F*. Thus, the *h*-b-ideal *M*_*m*_∗*B*∗*G*_*m*_ ∈ *B*_*m*_(*H*). Furthermore, *B*_*m*_(*H*) be a subsemigroup of *B*(*H*). As a result, *B*_*m*_(*H*) is bi-ideal of *B*(*H*). For some *M*_*m*_ ∈ *B*_*m*_(*H*), let us assume the *h*-bi-ideal *M*_*m*_∗*M*_*m*_. Then, $M_{m}*{\text{M}}_{m}=\overset{¯}{M_{m}M_{m}}\subseteq \overset{¯}{M_{m}}=M_{m}$ and minimality of *M*_*m*_ shows that *M*_*m*_∗*M*_*m*_ = *M*_*m*_. Since, also, *M*_*m*_∗*M*_*m*_∗*M*_*m*_ is *h*-bi-ideal, from $M_{m}*M_{m}*M_{m}=\overset{¯}{M_{m}BM_{m}}\subseteq M_{m}$ and minimality of *M*_*m*_ it means that *M*_*m*_∗*B*∗*M*_*m*_ = *M*_*m*_.

## 6. Conclusion

This research represents *h-*regular semiring along their *h*-ideals. The different subclasses of the *h*-regular semiring are described by their *h*-bi-ideal semigroup. We have shown that *B*(*H*) = *ℛ*(*H*)*ℒ*(*H*) for *h*-regular semiring *H*. We have characterized a new class of semigroup of *h-*bi-ideals in *h*-Clifford semiring. Lastly, we worked on minimal *h-*ideal along their *h-*bi*-*ideals and proved that *B*_*m*_(*H*) is a rectangular band. This research further can be extended with *h*-quasi ideals and *k*-ideals. The other idea of its extension is in the field of biology by using in growth-fragmentation-coagulation equation.

The article "Some Study of Semigroups of h-Bi-Ideals of Semirings" was retracted in 2023. Reasons: suspected computer-generated content; unreliable results or conclusions; concerns about the data; concerns about the results or conclusions.

## Data Availability

No data were used in this research.
